RETRACTED

# Increased Gut Redox and Depletion of Anaerobic and Methanogenic Prokaryotes in Severe Acute Malnutrition

**DOI:** 10.1038/srep26051

**Published:** 2016-05-17

**Authors:** Matthieu Million, Maryam Tidjani Alou, Saber Khelaifia, Dipankar Bachar, Jean-Christophe Lagier, Niokhor Dione, Souleymane Brah, Perrine Hugon, Vincent Lombard, Fabrice Armougom, Julien Fromonot, Catherine Robert, Caroline Michelle, Aldiouma Diallo, Alexandre Fabre, Régis Guieu, Cheikh Sokhna, Bernard Henrissat, Philippe Parola, Didier Raoult

**Affiliations:** 1 Aix-Marseille Université, Unité de Recherche sur les Maladies Infectieuses et Tropicales Emergentes, UM63, CNRS 7278, IRD 198, INSERM 1095, Marseille, France; 2 Hôpital National de Niamey, Niamey, Niger; 3 Centre National de la Recherche Scientifique, UMR 7257, 13288 Marseille, France; 4 Aix-Marseille Université, Architecture et Fonctions des Macromolécules Biologiques, 163, avenue de Luminy, 13288 Marseille cedex 9, France; 5 Laboratoire de Biochimie, hôpital de la Timone, UMR MD2, IRBA, Marseille, France; 6 Institut de Recherche pour le Développement (IRD), URMITE, Dakar, Sénégal; 7 Service de pédiatrie multidisciplinaire, hôpital de la Timone Enfant, APHM, Marseille France; 8 UMR_S 910, Aix-Marseille Université, Marseille, France; 9 Department of Biological Sciences, King Abdulaziz University, Jeddah, Saudi Arabia

## Abstract

Severe acute malnutrition (SAM) is associated with inadequate diet, low levels of plasma antioxidants and gut microbiota alterations. The link between gut redox and microbial alterations, however, remains unexplored. By sequencing the gut microbiomes of 79 children of varying nutritional status from three centers in Senegal and Niger, we found a dramatic depletion of obligate anaerobes in malnutrition. This was confirmed in an individual patient data meta-analysis including 107 cases and 77 controls from 5 different African and Asian countries. Specifically, several species of the *Bacteroidaceae*, *Eubacteriaceae*, *Lachnospiraceae* and *Ruminococceae* families were consistently depleted while *Enterococcus faecalis*, *Escherichia coli* and *Staphylococcus aureus* were consistently enriched. Further analyses on our samples revealed increased fecal redox potential, decreased total bacterial number and dramatic *Methanobrevibacter smithii* depletion. Indeed, *M. smithii* was detected in more than half of the controls but in none of the cases. No causality was demonstrated but, based on our results, we propose a unifying theory linking microbiota specificity, lacking anaerobes and archaea, to low antioxidant nutrients, and lower food conversion.

Malnutrition is estimated to cause 3 million child deaths annually or 45% of all child deaths^1^ and reflects the first Millennium Development Goal^2^. Severe acute malnutrition (SAM) is defined as a very low weight-for-height z-score (WHZ < −3 SD, corresponding to a weight below the average weight of healthy controls of the same height minus 3 standard deviations calculated according to World Health Organization (WHO) standards^3^), a mid-upper-arm circumference (MUAC) of less than 115 mm in children aged 6–59 months, or bilateral nutritional edema^2^. Its prevalence is estimated at 29 million children under 5 years of age^2^,^4^. SAM has been associated with high mortality (10–30%) and increased risk of diarrhea, pneumonia and systemic infections including bacteremia with *Staphylococcus aureus*, *Streptococcus*, *Salmonella*, *Klebsiella*, and *Escherichia coli*.

RETRACTED

SAM is not only associated with inadequate quantitative intake of energy and protein but also with a qualitative lack of micronutrients. The diet is restricted to cooked but contaminated starchy foods (rice, millet, sorghum) and lacks milk, meat, leafy vegetables and fruits (mango, orange, guava), which are natural sources of micronutrients and dietary antioxidants (vitamins A, C, E)^5^,^6^,^7^,^8^. This inadequate diet leads to low levels of antioxidants^9^, including uric acid, ascorbic acid^10^ and glutathione^11^, in the plasma and liver of these children. The resulting oxidative stress^12^ is a key feature in the pathophysiology of complicated (edematous) SAM^11^, confirmed through the beneficial effects of antioxidants^13^. However, only glutathione and alpha-lipoic acid supplementation have been shown to have positive effects on survival, while N-acetylcysteine, riboflavin, vitamin E and selenium were not shown to have a statistically significant effect^13^,^14^. Ready-to-use therapeutic food (RUTF), including several antioxidants, has recently revolutionized the management and prognosis of SAM in outpatient settings for children >6 months of age, without complications^15^, suggesting that the redox status could be altered in malnutrition.

Age, diet, and geography were first identified as major determinants of the gut microbiota^16^. While the link between gut microbiota and malnutrition has long been suspected, studies using metagenomic methods have revealed that specific gut microbiota alterations predict therapeutic failure^17^. In addition, gut microbiota immaturity persists despite therapeutic foods^18^. A recent review evidenced that the early depletion in gut *Bifidobacterium longum* represents the first step in gut microbiota alteration associated with severe acute malnutrition (SAM) before a disruption of the Healthy Mature Anaerobic Gut Microbiota (HMAGM), leading to diarrhea, malabsorption, deficient energy harvest and vitamin biosynthesis, and systemic invasion by microbial pathogens^19^.

RETRACTED

Archaea are typical representatives of the HMAGM worldwide^16^. Unlike the broad diversity of Bacteria in the gut, the Archaea comprised mainly members of the *Methanobacteriales* order, which are H2-oxidizing methanogens with *Methanobrevibacter smithii* being the leading representative species in healthy volunteers^20^. Significantly higher numbers of H2-utilizing methanogenic Archaea were observed in obese individuals than in normal-weight or post-gastric-bypass individuals leading to the hypothesis that interspecies H2 transfer between bacterial and archaeal species increases energy uptake by the human large intestine in obese persons^21^. As Archaea are vulnerable to trace amounts of free radicals, surviving only in a strongly reduced environment (redox potential < −200mV^22^), and, as such, are defined as extremely oxygen-sensitive prokaryotes, we hypothesized that a gut redox alteration, expected in SAM, should result in a major change in *Methanobrevibacter smithii* concentrations in the gut of severely undernourished children.

In this study, we tested whether gut obligate anaerobes are prone to depletion and determined whether aerotolerant species are prone to enrichment in the guts of severely undernourished children. We confirmed the putative depletion of extremely oxygen-sensitive prokaryotes, specifically targeting *Methanobrevibacter smithii*, representing the host-bacterial-archaeal mutualism^23^. We also analyzed the gut redox potential as a first step linking the lack of antioxidant and altered redox status, previously reported in malnutrition, to gut microbiota alterations. The confounding role of age^16^,^18^ was specifically ruled out through a sensitivity analysis including a matched-pairs study and meta-regression.

## Results

### Recruiting center bias

We screened 86 West African children of varying nutritional status (Dataset 1) and sequenced the fecal metagenome of 79 children from Dakar, Dielmo and N’Diop in Senegal and from Niamey in Niger. The samples from 10 children associated with a poor sequencing depth (<100,000 reads) were excluded and all other 69 samples were normalized to a 100,000 reads depth. To explore factors impacting gut microbial diversity among these 69 children with comparable gut metagenomes, we first performed a Pearson exploratory principal component analysis including relative abundances of the 2,245 identified bacterial species as active variables and center of recruitment, age, sex, and nutritional status as supplementary (explanatory) variables. Recruiting center alone differentiated children into distinct groups (Fig. 1), suggesting that geography is the main explanatory variable of overall gut microbiota variability. In a sensitivity analysis to test the robustness of our results, a second PCA was performed excluding 10 outliers (6 healthy children and 2 children with SAM from Dakar, Senegal, and 2 children with SAM from Niger) identified by the ROUT method^24^ (Q = 1%) based on the Euclidian distance to the framework origin (Supplementary Figure 1). This second PCA confirmed geography as the major determinant of the global variability of the gut microbiota among our samples. Strikingly, the children from Dielmo and N’Diop (south of Senegal, green) clustered with those of Niamey (Niger, red) at 2,124 km apart, but not with those from Dakar (Senegal, blue), which were much closer at 160 km. This dramatic center bias suggests that cases and controls should be recruited from the same center (and not only the same country) to identify gut microbiota alterations associated with any disease (malnutrition) and that multicenter data should not be pooled but require meta-analysis. Age, sex or nutritional status were not satisfactory explanatory variables of overall gut microbiota variability. As no children with SAM from Dielmo and N’Diop were included, these centers were excluded from subsequent analyses.

RETRACTED

### Gut microbiota maturation is associated with an enrichment in obligate anaerobes

After identifying the recruiting center bias and the need for meta-analysis, we sought to identify whether age has a significant impact on the enrichment or depletion of anaerobic bacteria in the digestive tract. Meta-regression appeared as the most suitable approach to identify whether age (gut microbiota maturation) was associated with enrichment or depletion of obligate anaerobes independently of nutritional status and recruiting center. We also decided to only include children with severe acute malnutrition (SAM) and healthy controls (CTL), strictly based on the WHO anthropometric criteria^2^,^3^, in order to improve the consistency among studies and to increase the power of the meta-analysis. Consequently, all children with other forms of malnutrition (moderate wasting, moderate to severe underweight and moderate to severe stunting) were excluded from this analysis.

After strict ascertainment of cases and controls, 10 cases and 11 controls from Dakar, Senegal and 10 cases and 9 controls from Niamey, Niger were included in 2 distinct comparisons in our meta-analysis. We also used this meta-analysis to test whether our results were similar to those of the published case-control studies with publicly available metagenomic data. Preliminary searches identified 26 records focusing on gut microbiota alterations associated with malnutrition; 21 records were immediately excluded however (Fig. 2). Thus, 5 full-text articles were assessed for eligibility, and 2 articles were further excluded because the assignment of metagenomics reads could not be obtained at the prokaryotic species level^25^,^26^. Consequently, our two comparisons, along with three comparisons from the literature^17^,^18^,^27^ were included from 5 different countries (Bangladesh, India, Malawi, Niger and Senegal) corresponding to 264 children (Table 1). After case and control ascertainment, only 107 children with SAM and 77 controls were included. Although individual assessment could not be performed for one study^18^, the risk of bias was considered to be low; therefore, these participants were included (Table 1).

RETRACTED

Our 2 comparisons and 2 of the 3 included comparisons from the literature were consistent with a positive summary aerotolerant odds ratio (AOR = (aerotolerant prokaryotes enriched in SAM x obligate anaerobic prokaryotes depleted in SAM)/(aerotolerant prokaryotes depleted in SAM x obligate anaerobic prokaryotes enriched in SAM), see methods) suggesting a relative depletion of obligate anaerobes and enrichment of aerotolerant organisms in SAM (AOR 5.00, 95% confidence interval (95%CI) 0.82–30.49, p = 0.08, Fig. 3a). Heterogeneity was however substantial (I^2^ = 81%) and significant (p = 0.0003), with one contradictory study^17^, prompting the detection of explanatory covariates. As suspected based on the literature^16^, meta-regression revealed that the age difference between cases and controls significantly altered the aerotolerant odds ratio (slope −0.06, 95%CI −0.12 to −0.0003, p = 0.048, Fig. 3b). Indeed, this confirmed that gut microbiota maturation is associated with an enrichment in obligate anaerobes^16^.

### Relative gut anaerobic depletion and aerotolerant enrichment in SAM

To check for the confounding role of age, we identified ten matched pairs, including six matched pairs in the Dakar study, along with two twin pairs from the Smith *et al*. study^17^. Strikingly, in this study, 9/11 ‘healthy’ co-twins presented severe stunting and did not fulfill our control selection criteria, so these pairs were excluded. Two matched pairs from the Ghosh *et al*. study^27^ were also included (Supplementary Table S1). Pairing was perfect for sex and highly effective for age (rs (Spearman) 0.98, p < 0.0001). The mean age ± SD was 20.3 ± 17.3 and 19.2 ± 15.3 for cases and controls, respectively (Wilcoxon matched-pairs signed rank test, p = 0.43), so that the confounding role of age was excluded, as the controls were slightly younger than cases, and obligate anaerobes increased with age^16^.

RETRACTED

The meta-analysis of these ten matched pairs, and participants of the Subramanian study (ruling out the confounding role of age using a linear mixed model, see Supplementary Table 15a of^18^), revealed a significantly increased AOR (10.59, 95%CI 2.17–51.69, p = 0.004). A subgroup analysis by continent reduced heterogeneity between studies (I^2^ reduced from 75% to 0%) with a significant subgroup difference (I2 = 91.3% − p = 0.0007, Fig. 3c). The direction of the effect was consistent in all four comparisons after ruling out the confounding roles of age, sex and bias associated with geography. These results suggest that SAM is associated with a dramatic relative anaerobic depletion regardless of age, sex and recruitment center (geography). Moreover, this relative anaerobic depletion may be more profound in Asia than in Africa.

The number of depleted anaerobes was several times higher than the number of enriched aerotolerant species in SAM in all comparisons [2.8 in Dakar (present study), 2.4 in India^27^, 2.9 in Malawi^17^ and 9.3 in Bangladesh^18^], suggesting that malnutrition was more closely associated with decreased anaerobic than increased aerotolerant diversity. A qualitative meta-analysis confirmed the depletion of several obligate anaerobes, including several *Firmicutes* (3 *Eubacteriaceae*, 3 *Lachnospiraceae*, 2 *Ruminococcaceae, 1 Erysipelotrichaceae), Bacteroidetes* (2 *Bacteroidaceae) and Actinobacteria (2 Eggerthella, 1 Coriobacteriaceae). Conversely*, some aerotolerant bacteria were enriched in SAM, including *Enterococcus faecalis, Escherichia coli*, and *Staphylococcus aureus*, which all represent potential pathogens (Fig. 4).

### Gut microbial and M. smithii depletion and increased redox potential in SAM

To clarify whether only relative, or also absolute abundance of obligate anaerobes, was depleted in SAM, we quantified the total bacterial number by flow cytometry. *M. smithii*, as one of the most oxygen-sensitive prokaryotes in the gut, was also assessed by quantitative real-time PCR to confirm anaerobic depletion. Redox potential was investigated in the fecal samples as a putative explanatory variable representing oxidation of the gut environment. The total bacterial concentration was significantly decreased in SAM (mean ± SD, 10.9 ± 0.30 log10 bacteria/g of stool in SAM versus 12.12 ± 0.42 in controls, two-tailed paired t-test p = 0.008, Fig. 5). With the aforementioned results, this confirmed the absolute decrease in gut obligate anaerobes in SAM. This was further confirmed by the fact that *M. smithii* was detected in five out of six controls but not in the cases (McNemar test, p = 0.04). Gut redox was abnormally positive and significantly increased in SAM (mean ± SD (mV), 27.0 ± 47.8 vs. −26.5 ± 61.8, p = 0.001).

RETRACTED

Including all participants from Niger and Senegal, *M. smithii* was not detected in the 20 children with SAM, although this microbe was detected in 40% and 75% of controls (p < 10^−4^) based on v3v4 16S rRNA large-scale sequencing and qPCR, respectively (Supplementary Table S2). We compared all cases and ascertained controls recruited in Dakar in a linear regression model, with age, sex, and SAM as the independent variables. Finally, SAM was the only independent predictor of the total bacterial count (SAM, −0.78, −1.31 to −0.25, p = 0.007 – R^2^ = 0.39), *M. smithii* concentration (−4.28, −6.41 to −2.15, p = 0.0004, R^2^ = 0.47) and fecal redox potential (coefficient 51.38, 0.71 – 102.05, p = 0.047, R^2^ = 0.20).

## Discussion

In the present study, we observed global bacterial depletion, a depletion in obligate anaerobes and a lack of methanogens in the gut microbiota of children with SAM. Quantifying the fecal redox potential as an explanatory parameter, we found for the first time a gut environment oxidation associated with childhood SAM. We identified the depletion of many oxygen-intolerant prokaryotes, while a small number of aerotolerant and potentially pathogenic prokaryotes were enriched in the gut of children with SAM. In particular, the well-known potential pathogens *Enterococcus faecalis*, *Escherichia coli* and *Staphylococcus aureus* were consistently enriched in SAM while *Methanobrevibacter smithii*, the prokaryote most sensitive to oxygen and the main representative of Archaea in the gut^20^, was not detected in children with SAM. These results found in two West African centers (Niger and Senegal) were reproduced by reanalysis of previously published studies^17^,^18^,^27^ from different countries (Bangladesh, India and Malawi) and different continents (Africa and Asia). Using principal component analysis and meta-analysis, the geographical bias^16^ was confirmed and controlled for. Using matched-pairs, meta-regression, and multivariate linear regression analyses, the confounding role for age^16^,^18^ was confirmed and controlled for.

The results of our study led us to propose a unifying theory linking gut environment oxidation to depletion of anaerobic and methanogenic prokaryotes in severe acute malnutrition^28^. The lack of adequate breastfeeding and nutrients^5^,^6^,^29^, maintaining the natural fecal anti-oxidant capacity^30^, is the most probable cause. Indeed, as a diet selected to raise the intake of dietary antioxidants increases the fecal antioxidant capacity^30^,^31^,^32^,^33^, a diet depleted in antioxidants, as previously reported in SAM^6^, is expected to decrease the fecal antioxidant capacity.

RETRACTED

Abnormal inversion of the ratio of anaerobes to aerobes has been reported for a long time in SAM, with incomplete correction after treatment^19^,^34^. *In vitro*, antioxidants are able to keep highly oxygen-sensitive bacteria alive in ambient air^35^ and facilitate the *in vitro* aerobic culture of *Bacteroides*^36^. In humans or in a batch-culture fermentation system reflective of the distal region of the human large intestine, flavonoids, with a 3–5 times greater antioxidant capacity than vitamins C or E *in vitro* and being poorly absorbed in the gut^37^,^38^, dramatically increase microbial members of the HMAGM^16^,^19^ including *Eubacterium rectale*^16^ and *Blautia coccoides*^39^,^40^. Strikingly, *Eubacterium rectale* was found consistently depleted in SAM (Fig. 4). HMAGM maintenance by antioxidants could also explain why glutathione dramatically reduces *Helicobacter*-induced gastric pathologies^41^.

Host-bacterial-archeal mutualism was recently demonstrated as a key in improving food conversion (the mass of food eaten divided by the weight gain): In gnotobiotic animals, gut colonization by the anaerobe *Bacteroides thetaiotaomicron* increased food conversion limited by H2 accumulation^23^. Cocolonization by *B. thetaiotaomicron* and *M. smithii* resulted in optimal food conversion via the removal of the H2 excess by methanogenesis^23^. While this process was considered to be impossible in ambient air, we recently demonstrated that bacteria considered unable to grow in aerobic atmospheres (anaerobic), are indeed able to grow in such an environment provided that the medium contains adequate antioxidants^36^. Moreover, we were also able to produce methane (methanogenesis) by *B. thetaiotaomicron* and *M. smithii* in aerobic atmosphere using ascorbate, uric acid and gluthatione^42^. This experimental evidence led us to suspect a causal link between the lack of dietary antioxidants, anaerobic depletion (including *B. thetaiotaomicron* and *M. smithii*), and decreased energy harvest and food conversion.

Despite the reported associations and *in vitro* experimental model, no definite evidence for a causal role of diet or gut redox on anaerobic depletion is presented and other factors should be discussed. Age, determining gut colonization by obligate anaerobes^16^,^18^ and methanogens including *M. smithii*^16^,^18^,^20^, was controlled for using matched-pairs and multivariate linear regression analyses. Diet is not the only factor as human submucosal gland secretions contain uric acid that serves as an antioxidant^43^. A contaminated environment may play a role through injection of pathogens in the gut microbiota. Subsequent proliferation of pathogens in the gut in association with gut microbiota alteration could result in a host disease defined as a ‘gut microbiota infection’^44^. Among such pathogens, *Salmonella enterica* and *Clostridium difficile* pathogenic strains have been shown to deplete the global and more specifically the anaerobic gut microbiota, regardless of diet^45^,^46^. Other factors able to deplete gut anaerobes include the lack of nutrients devoid of antioxidants but shaping the gut microbiota (prebiotics^47^), host genetic factors^48^, altered innate lymphoid cells^49^ and deficient fucosylation^50^. Here, we propose that gut redox is a key parameter shaping the gut microbiota. The relative role of gut redox alteration among all factors influencing the gut microbiota (including intestinal inflammation, which itself could alter the gut redox) will be elucidated by future studies.

RETRACTED

Our findings provide new and important insights into the vicious cycle of malnutrition, correlating altered redox metabolism with a possibly irreversible disruption of host-archaeal-bacterial mutualism, via a depletion of anaerobes and methanogens. Parallel invasion by aerotolerant bacterial pathogens highlights the need for antibiotics as previously demonstrated^51^. Additional studies are needed to confirm the oxidation of the gut environment in SAM and to test the beneficial effect of RUTF and antioxidants in the restoration of gut obligate anaerobes and methanogens. Different antioxidants may have different effects^13^,^14^ with no effect of antioxidants completely absorbed in the proximal gut^52^ or not associated with adequate breastfeeding, nutrition and gut microbiota infection control. Based on our results, new therapeutic options could be tested in severe or refractory SAM cases in association with antibiotics and up-to-date management^15^, including higher levels of antioxidants, unabsorbed antioxidants (carotenoids and flavonoids)^37^, supplementation of lacking microorganisms and transplantation of fecal microbiota.

## Materials and Methods

### Experimental design

We conducted two prospective case-control studies in Niger (Niamey) and Senegal (Dakar, Dielmo (13°43′N 16°24′W) and NDiop (13°41′N 16°22′W)). Dielmo and N’Diop are two contiguous villages included in a longitudinal malaria survey^53^. The gut microbiota of children with varying nutritional status were analyzed using a principal component analysis before comparing children with SAM (according to the 2009 WHO criteria^2^,^3^) to ascertained healthy controls (CTL) according to the STROBE statements^54^. Recruitment of children <60 months attending the clinic ‘Notre Dame de L’Esperance’ for malnutrition in Thiaroye, Dakar, Senegal, occurred in April, 2014. Children from Dielmo and Ndiop were recruited between September and December 2014 and recruitment of children from the National Hospital, Niamey, Niger ranged from February to November 2014. The exclusion criteria included the following: absence of parent or patient consent, antibiotic administration <2 months before stool collection and insufficient fecal amount. Exclusion criteria for controls included any form of malnutrition, presence of fever, acute respiratory infection (cough), acute or chronic diarrhea in the previous 4 weeks. Symptoms and complications of malnutrition (cough, fever, diarrhea, vomiting), or other forms of malnutrition (moderate to severe stunting and underweight) were not a reason for exclusion for cases since they are considered as a direct consequence and part of severe acute malnutrition. Clinical data (sex, date of birth, date of sampling, clinical history, weight, height, mid-upper arm circumference and antibiotic use) were recorded using a standardized questionnaire. Growth monitoring parameters (weight-for-length (WHZ), weight-for-age (WAZ) and height-for-age (HAZ) z scores) were assessed using the WHO Anthro v3.2.2, January 2011. Length was measured recumbently for children less than 12 months of age and height was measured standing in children greater than 12 months of age. WHZ and WAZ, however, are not appropriate in the presence of edematous SAM. After collection using sterile plastic containers, the stool samples were aliquoted and frozen at −80 °C until manipulations.

RETRACTED

All aspects of the study were approved by the local ethics committee ‘Comité d’éthique de l’IFR 48, Service de Médecine Légale (Faculté de Médecine, Marseille, France) under accession number 09–022, 2010. Informed consent was obtained and the nature and possible consequences of the studies were explained. Only verbal consent from patients or parents was required for this study according to French bioethics decree Number 2007–1220, published in the official journal of the French Republic and to article L1211-2 of the French Code of Public Health. Professor DIALLO and Professor ADEHOSSI certified that this study was not in opposition to the declaration of Helsinki and in accordance with Senegalese and Nigerien laws respectively (certificates available on request).

### Case and control definition and ascertainment

Cases were children with SAM defined as a WHZ <−3 standard deviations (SD), calculated according to WHO standards, a MUAC of less than 115 mm in children aged 6–59 months, or bilateral nutritional edema^2^,^3^. Control children were asymptomatic (no cough, fever, diarrhea or vomiting) without any form of malnutrition (WHZ > −2 SD, Height-for-age Z-score >−2 SD, weight-for-age z-score >−2 SD, MUAC >125 mm in children aged 6–59 months) attending the centers for non-nutritive disorders. Local nutritional experts (AD, SB) performed the case ascertainment and control selection, and the clinical and anthropometric data were verified (MM).

RETRACTED

### Treatment of undernourished children

None of the undernourished children were in feeding programs prior to hospital admission. Fecal sampling preceded anti-infectious treatment in all cases. In Senegal, an energetic milk (milk, oil, sugar) was given immediately along with amoxicillin, most often in connection with a skin infection. An Emmel test (HbS detection), a thick smear, and a direct stool parasitological examination were systematically performed. Specific treatment was given based on the results (Artemisinin-based combination therapy, mebendazole and/or metronidazole), but none of the included children were found to be positive for parasites. Vitamin A was given only after stabilization, always after fecal sampling. If complicated malnutrition was diagnosed, the child was referred to the University Hospital. In Niger, children were recruited immediately on diagnosis, before any treatment or lipid-based nutritional supplements was administered. Self-medication was also excluded, so that bias in reporting of antibiotic administration <2 months before stool collection was minimized. Overall, the anti-anaerobic effect of anti-infectious drugs (metronidazole), frequently used in the malnutrition setting, played no confounding role in this study.

### Outcomes, exposure and predictors

The principal summary measure was the ‘aerotolerant’ odds ratio (AOR), calculated as follows: AOR = (number of aerotolerant species enriched in SAM × number of obligate anaerobes depleted in SAM)/(number of aerotolerant species depleted in SAM × number of obligate anaerobes enriched in SAM).

### Sequencing and biochemical methods

Sequencing was performed using 16S v3v4 amplification prior to large-scale sequencing using an Illumina MiSeq Engine. Assignment was performed down to the species level. To control for depth bias, samples yielding less than 100,000 reads at the species level were subsequently excluded prior to the normalization of the remaining samples (all relative abundance <10^−5^ were converted to 0). Specific PCR analyses targeting *M. smithii* were performed as previously described^20^. Fecal redox was measured, and total bacterial concentration was assessed using flow cytometry (methods are fully detailed in Supplementary Data).

RETRACTED

### Database of obligate anaerobes

A bacterial oxygen tolerance database was generated based on the literature (Supplementary Methods, available online at http://www.mediterranee-infection.com/article.php?laref=374). Each phylotype was assigned as ‘obligate anaerobe’, ‘aerotolerant’ or ‘unknown’ according to oxygen tolerance.

### Statistical analysis

After normalization, an exploratory Pearson principal component analysis was first performed using the relative abundance of bacterial species as active variable and age, sex, and nutritional status as supplementary elements using XLSTAT v2014.3.07 (Addinsoft, Paris, France). The ROUT method (Q = 1%)^24^ was used to robustly identify outliers based on the Euclidian distance to the framework origin (PCA centroid) calculated using the first three components of each sample. Thus, in each center, species were considered to be enriched or depleted in cases or controls based on univariate linear regression calculated using MINE^55^ with the R package version 3.1.0. Pairing was conducted to control for age and sex, selecting cases and controls with the same sex, center recruitment and closest age. A paired t-test and McNemar test were used to compare the total number of bacteria, fecal redox potential and presence of *M. smithii* between age- and sex-matched pairs, respectively. Different multivariable stepwise linear regression models were created, including either total bacterial concentration, *M. smithii* concentration or fecal redox potential as the dependent variable and age, sex and SAM as the independent variables using SPSS v24.0 (IBM, Paris, France). All tests were two-sided, and a p-value < 0.05 was considered significant.

### Meta-analysis of individual patient data

We performed a meta-analysis of individual patient data with meta-regression controlling for age according to the MOOSE guidelines^56^ including our two comparisons (Dakar (Senegal) and Niamey (Niger) – no children with SAM were recruited in Dielmo & N’Diop). Eligibility criteria for other studies included analyzing the fecal prokaryotes of children with SAM and healthy controls using metagenomic methods at the species level. The search terms included severe acute malnutrition, kwashiorkor, marasmus AND metagenome or microbiota. There was no restriction according to date or language. The selection and ascertainment criteria for the cases and controls were applied as described above when individual data were available. The protocols (PICOS), exclusion criteria, data preparation and bias assessment are detailed in the Supplementary Methods and Supplementary Table S3. The meta-analysis was performed using the Mantel-Haenszel method and a random-effects model using Review Manager version 5.2 (Cochrane Collaboration, Copenhagen, Denmark). Heterogeneity was assessed using I^2^ analysis. Meta-regression controlling for age was performed using comprehensive meta-analysis version 2.2.064 (Biostat, Englewood, NJ, USA) as reported by Borenstein *et al*.^57^.

RETRACTED

## Additional Information

**Accession codes:** Metagenomic datasets have been deposited at the EBI (http://www.ebi.ac.uk/) under accession codes PRJEB7053.

**How to cite this article**: Million, M. *et al*. Increased Gut Redox and Depletion of Anaerobic and Methanogenic Prokaryotes in Severe Acute Malnutrition. *Sci. Rep*. **6**, 26051; doi: 10.1038/srep26051 (2016).

## Supplementary Material

Supplementary Information

Supplementary Data

## Figures and Tables

**Figure 1:** Explanatory variables of global variability of the 16S rRNA gut microbiota among 69 West African children of varying nutritional status. (**a**) A Pearson Principal component analysis (PCA) of the 16S rRNA gut metagenomes of 69 West African children revealed that geography was the main factor in gut microbiota variability, as only recruiting centers differentiated children into distinct groups (up). (**b**) In a sensitivity analysis to test the robustness of the results, a second PCA was performed excluding 10 outliers (6 healthy children and 2 children with SAM from Dakar, Senegal, and 2 children with SAM from Niamey, Niger) identified by the ROUT method (Q = 1%) based on the Euclidian distance to the framework origin^24^. This second PCA confirmed geography as the major determinant of the global variability of the gut microbiota among our samples (down). *City*: blue: Dakar (Senegal), green: Dielmo and N’Diop (contiguous villages in Senegal), red: Niamey (Niger). *Age*: red: up to 12 months, blue: >12 months and up to 24 months, green: >24 months, grey: missing data, *Sex*: red: female, blue: male, *Nutritional status*: green: healthy controls, red: severe acute malnutrition, blue: children with other forms of malnutrition.

**Figure 2:** Meta-analysis study flow diagram. A literature review of case-control studies with available metagenomic data at the species level identified 5 comparisons eligible for meta-analysis. Study selection was performed according to the MOOSE checklist and guidelines. The 2 excluded full-text articles were studies from Monira^25^ and Gupta^26^.

**Figure 3:** Meta-analysis of all ascertained cases and controls. A positive aerotolerant odds ratio (AOR) correspond to a relative aerotolerant enrichment/anaerobic depletion in SAM. (**a**) Before controlling for age, there was a trend for an increased AOR in severe acute malnutrition (SAM), but heterogeneity was substantial, (**b**) Meta-regression confirmed that age difference between cases and controls significantly altered the AOR. (**c**) Matched pairs analysis (mixed linear regression for Subramanian controlling for age) found a dramatic and significant anaerobic gut prokaryote depletion in SAM independently of geography and age. SAM: severe acute malnutrition, BGD: Bangladesh.

RETRACTED

**Figure 4:** Species consistently enriched and/or depleted in SAM. Qualitative meta-analysis identified the depletion of several obligate anaerobes and an enrichment of the aerotolerant *Enterococcus faecalis*, *Escherichia coli* and *Staphylococcus aureus* in SAM. Red: enriched in SAM. Green: depleted in SAM. *Potential human pathogens. SAM: severe acute malnutrition, LAB: Lactic acid bacteria.

**Figure 5:** Alteration of gut total bacterial number, *M. smithii* and redox potential in SAM. (**a**) Two-sided paired t-test. (**b**) McNemar test. Total gut bacterial concentration and *M. smithii* were significantly depleted in SAM while the gut redox potential was increased in SAM. These results, obtained after analysis of 6 age- and sex-matched pairs, were confirmed by a linear regression model including all 21 individuals from Dakar, Senegal with age, sex and SAM as the independent variables. SAM: severe acute malnutrition, CTL: healthy controls.

**Table 1:** Studies comparing the gut metagenomes of children with severe acute malnutrition to healthy controls.

Reference	Dates	Country, city, center	Study design	Method of fecal metagenomics analysis, sequencing depth	Number of screened children (number of 16S metagenomes)	Individual data available	Number of ascertained SAM cases included in the meta-analysis (nb of 16S metagenomes)	Number of ascertained controls included in the meta-analysis (nb of 16S metagenomes)
Present study, Niger	2014	Niger, Niamey	Observational study	V3v4 Illumina MiSeq, 200,000 reads	34 (28)	Yes	10 (10)	9 (9)
Present study, Senegal	2014	Senegal, Dakar	Observational study	V3v4 Illumina MiSeq, 200,000 reads	52 (51)	Yes	10 (10)	11 (11)
Smith^17^	2013	Malawi, Southern region, 5 centers (Mayaka, Mbiza, Chamba, Mitondo, Makhwira)	longitudinal comparative study of monozygotic and dizygotic twin pairs	V4 16S Illumina HiSeq instrument, 116,414 reads	44 (183)	Yes	14 - Mayaka 3, Mbiza 3, Chamba 4, Mitondo 1, Makhwira 3 –(15)	5 - Mbiza 4, Chamba 1 (6)
Subramanian^18^	2014	Bangladesh, Dhaka	Cohort study	V4 16S Illumina HiSeq instrument, unknown metagenomics depth	114 (1074)^a^	No but species enriched or depleted in SAM calculated using a mixed linear regression model controlling for age available in online supplementary material	64 (78)^a^	50 (996)^a^
Ghosh^27^	2014	India, Birbhum district	Observational studies of children with varying nutritional status	Untargeted sequencing GS-FLX, 10,000 reads^b^	20 (20)	Yes	9 (9)	2 (2)
Total					264 screened children (1356)		107 (122)	77 (1024)

^a^Information kindly communicated by the authors^18^.

^b^Raw data were reanalyzed by one of us (BD) to obtain species assignement (see supplementary methods). SAM: severe acute malnutrition.
